# Pollen Viability, Pistil Receptivity, and Embryo Development in Hybridization of *Nelumbo nucifera* Gaertn

**DOI:** 10.1100/2012/678706

**Published:** 2012-05-02

**Authors:** Yan-Li Wang, Zhi-Yong Guan, Fa-Di Chen, Wei-Min Fang, Nian-Jun Teng

**Affiliations:** College of Horticulture, Nanjing Agricultural University, Nanjing 210095, China

## Abstract

Seed set is usually low and differs for different crosses of flower lotus (*Nelumbo nucifera* Gaertn.). The reasons remain unknown, and this has a negative impact on lotus breeding. To determine the causes, we carried out two crosses of flower lotus, that is, “Jinsenianhua” × “Qinhuaihuadeng” and “Qinhuaihuadeng” × “Jinsenianhua” and pollen viability, pistil receptivity, and embryo development were investigated. The pollen grains collected at 05:00-06:00 hrs had the highest viability, and the viabilities of “Jinsenianhua” and “Qinhuaihuadeng” were 20.6 and 15.7%, respectively. At 4 h after artificial pollination, the number of pollen grains germinating on each stigma reached a peak: 63.0 and 17.2 per stigma in “Jinsenianhua” × “Qinhuaihuadeng” and “Qinhuaihuadeng” × “Jinsenianhua”, respectively. At 1 d after artificial pollination, the percentages of normal embryos in the two crosses were 55.0 and 21.9%, respectively; however, at 11 d after pollination, the corresponding percentages were 20.8 and 11.2%. Seed sets of the two crosses were 17.9 and 8.0%, respectively. The results suggested that low pistil receptivity and embryo abortion caused low seed set in “Qinhuaihuadeng” × “Jinsenianhua”, whereas low fecundity of “Jinsenianhua” × “Qinhuaihuadeng” was mainly attributable to embryo abortion.

## 1. Introduction

The lotus (*Nelumbo nucifera* Gaertn.) is an economically important aquatic plant in the family of Nelumbonaceae. In general, lotus is grouped into three categories based on utilization and morphological features: rhizome lotus, seed lotus, and flower lotus. Lotus has been cultivated for more than 2000 years in China and its current cultivation area covers most parts of China [1–3]. The flower lotus is one of the ten most famous traditional flowers in China and is widely cultivated in gardens and scenic spots for environmental beautification and water purification [4–6]. As the Chinese economy, people's living standards and the tourism industry have rapidly improved in recent years, the flower lotus has played an increasingly important role in cleaning and beautifying the environment. Various breeding methods including artificial hybridization, radiation techniques, and multiploid approach have been applied to develop new lotus cultivars [6–8]. Among these methods, artificial hybridization is the most widely used and most effective way to produce new lotus cultivars. Although there have been some new lotus cultivars developed by traditional hybridization breeding in the past two decades in China, reproductive barriers often exist in artificial hybridization and seriously reduce the breeding efficiency of lotus [6]. To date, few studies have examined reproductive barriers in lotus hybridization, thus the factors affecting the breeding efficiency of flower lotus remain unknown.

Because the features of parental reproductive systems and the interaction of their systems are usually related to breeding efficiency in plant cross-breeding, thus the parental reproductive systems and reproductive behaviors after pollination have been extensively investigated in many plants, for example, *Dendranthema grandiflorum*,* Fragaria ananassa,* and *Phaseolus vulgaris* [9–11]. Many of these studies have successfully revealed the reasons leading to reduction in seed production and breeding efficiency. Enlightened by these previous studies, we carried out a systematic investigation of factors that may affect breeding efficiency of flower lotus in the present study. These factors included pollen viability of male parents just before artificial pollination, germination behavior of pollen grains on stigmas after artificial pollination, and embryo development after fertilization. The purpose of this study was to unravel the main factors causing low fecundity in the cross-breeding of water lotus. The expected output will provide valuable information for efficient measures to overcome reproductive barriers and improve breeding efficiency of water lotus and other crops, in the future.

## 2. Materials and Methods

### 2.1. Plant Materials

Two crosses of flower lotus (*N*.* nucifera*) were performed: “Jinsenianhua” (female plant) × “Qinhuaihuadeng” (male) and “Qinhuaihuadeng” (female) × “Jinsenianhua” (male). All plants were grown in Nanjing Yileen, Zhujiang Town, Pukou District, Nanjing, China (32°07′ N, 118°62′ E). In the past several years, we have carried out many lotus crosses and found that seed set was very low in some crosses. Therefore, two representative lotus cultivars were used for reciprocal crosses in the present study, aiming to reveal the factors affecting breeding efficiency of flower lotus.

### 2.2. Pollen Viability

Lotus pollen is usually viable for a few hours after shedding, and the viability is difficult to determine. We previously systematically investigated lotus pollen viability using different methods: fluorescein diacetate (FDA), triphenyltetrazolium chloride (TTC), germination in vitro, and the peroxidase method. The methods of FDA, TTC, and germination in vitro were not suitable for checking pollen viability, and so we used the peroxidase method. On sunny days, fresh pollen grains were, respectively, collected at 05:00-06:00 hrs, 06:00-07:00 hrs, and 07:00-08:00 hrs. The liquid for determining pollen viability comprised two reagents: reagent I (1 : 1 : 1 of 0.5% benzidine, 0.5% *α*-naphthol and 0.25% sodium carbonate) and reagent II (0.3% hydrogen peroxide solution). The pollen grains under test were distributed on a glass slide coated in the culture medium comprising one drop of each of reagents I and II and then incubated at 30°C for 30 min. The pollen grains stained red if they were viable, and viable grains were counted in ten optical fields (at least 50 pollen grains per field) under an Olympus BX41 microscope. Each experiment was repeated three times and statistical analysis was performed by Tukey's test.

### 2.3. Sexual Hybridization

 Lotus is an insect-pollinated species and its pistil matures 1-2 d before the stamens, thus we did not emasculate the flowers of female plants and only bagged them at 2 d before their pistils matured. When the female flowers opened and the stigmas were full of bright yellow mucus, this indicated the most suitable period for pollination. We carried out artificial pollination at 06:00–08:00 hrs on sunny days using fresh pollen collected from male plants at 05:00-06:00 hrs. The crosses were performed from late July to early August 2009, when average temperature was approximately 31°C, with range 26–38°C.

### 2.4. Pollen Germination on Stigmas after Artificial Pollination

Germination of pollen grains on stigmas was examined using the method of Sun et al. [11] with minor modifications. Thirty pistils were, respectively, sampled at 0.5, 1, 2, 4, 6, 8, 10, and 12 h after pollination and fixed and stored in FAA solution (5 : 5 : 90 of formalin, acetic acid and 70% ethanol) at 4°C until use. The samples were softened overnight in 1 mol L^−1^ NaOH, rinsed in water and mounted on a microscope slide with a drop of 0.1% aniline blue (0.1 mol L^−1^ K_3_PO_4_ supplemented with 18% glycerol), and then observed under a fluorescence microscope (Zeiss Axioskop 40; Carl Zeiss Shanghai Company Ltd, Shanghai, China) with excitation filter BP 395–440, chromatic beam splitter FT 460, and barrier filter LP 470. Digital images were captured using an Axiocam MRC camera [12]. In addition, some pistils were fixed in 2.5% glutaraldehyde (0.1 M phosphate buffer, pH 7.2). After rinsing in buffer, the samples were postfixed overnight in 1% (w*⁄*v) buffered osmium tetroxide, washed in buffer, dehydrated in an ethanol series (40, 70, 90 and 100%, 15 min each time), and then critical-point-dried using liquid CO_2_. The pistils were then mounted on aluminum specimen stubs with adhesive tabs. After coating with gold, they were examined using a Philips XL-30 environment scanning electron microscope (SEM) (Hitachi S-3000N) [13].

### 2.5. Embryo Development after Pollination and Seed Set

About 80 ovaries at 1 and 2 d after pollination were, respectively, collected and then immersed in FAA at 4°C until use for examination of embryo development. The ovules were dehydrated through a graded series of alcohol solutions (70, 85, 95, and 100%, 5 min each time), infiltrated with xylene, and embedded in paraffin wax [11]. Sections were cut to a thickness of 8–10 *μ*m using a Leica RM2016 microtome (Shanghai Leica Instruments Co Ltd, China), stained in Heidenhain's haematoxylin, and were observed and photographed under the Zeiss Axioskop 40 microscope. In addition, we collected about 80 ovaries at different periods after pollination in order to examine the percentage of normal embryos, and the samples were observed under a stereomicroscope equipped with a digital camera.

One month after artificial pollination, about 30 lotus seed pods were randomly chosen and plump seeds were collected from them. Then seed set in each cross was calculated with the following formula: seed set = (number of plump seeds/total number of pollinated stigmas) × 100% [11].

### 2.6. Statistical Analysis

The data were analysed by a one-way analysis of variance using the SPSS software 16.0 (SPSS Inc, Chicago, IL, USA). Tukey's Honestly Significant Difference (HSD) (*P* ≤ 0.05) was used to discriminate the values.

## 3. Results

### 3.1. Viability of Pollen Grains Collected at Different Times

 The collection time of lotus pollen grains significantly affected pollen viability (Figure 1): viabilities of “Jinsenianhua” pollen grains collected at 05:00-06:00 hrs, 06:00-07:00 hrs, and 07:00-08:00 hrs were 20.6, 12.1, and 6.8%, respectively; the corresponding values for “Qinhuaihuadeng” were 15.7, 7.7 and 5.4%. In addition, there was no significant difference in viabilities of pollen grains collected at 05:00-06:00 hrs between “Jinsenianhua” and “Qinhuaihuadeng”. Since pollen grains collected at 5:00-6:00 hrs had the highest viability for both cultivars, we therefore carried out artificial pollination experiments using pollen grains collected in this time span.

### 3.2. Pollen Germination on Stigmas after Artificial Pollination

In both crosses, some pollen grains germinated within 0.5 h of artificial pollination. After that, more pollen grains germinated on stigmas and the number reached a peak at 4 h after pollination (Table 1; Figures 2(A), 2(B)): there were on average 63.0 and 17.2 germinated pollen grains per stigma at 4 h after pollination in the crosses “Jinsenianhua” × “Qinhuaihuadeng” and “Qinhuaihuadeng” × “Jinsenianhua”, respectively. Then, at 12 h, the corresponding numbers of germinated pollen grains on each stigma gradually decreased to 13.8 and 7.4. Although the change pattern of the number of germinated pollen grains on stigmas was very similar for the two crosses, the number in the cross “Jinsenianhua” × “Qinhuaihuadeng” was significantly higher than that of “Qinhuaihuadeng” × “Jinsenianhua” at each time point after pollination (Table 1). Moreover, there were many pollen tubes with abnormalities such as branching, splitting, coiling, and convolution on stigmas in the “Jinsenianhua” × “Qinhuaihuadeng” cross, which resulted in the failure of these pollen tubes penetrating the stigma surface (Figures 2(C)–2(E)). In contrast, most pollen tubes grew normally and entered the stigma surface for “Jinsenianhua” × “Qinhuaihuadeng” (Figure 2(F)).

### 3.3. Percentage of Normal Embryos

Zygotes divided very quickly in the two crosses. For example, at 1 d after artificial pollination, globular embryos were observed in many ovules, and heart embryos were observed in some ovules at 2 d after artificial pollination (Figures 2(G), 2(H)). At 4 d after pollination, most embryos had reached the cotyledon embryo stage. Normal globular embryos were observed in 55.0% of ovaries at 1 d after pollination, and normal heart embryos were observed in 37.5% of ovaries at 2 d after pollination in the “Jinsenianhua” × “Qinhuaihuadeng” cross (Table 2). However, the corresponding values for the “Qinhuaihuadeng” × “Jinsenianhua” cross were 21.9 and 14.7%, respectively. As the embryos continued to develop, increasing numbers of embryos degenerated in the two crosses (Table 2; Figures 3(A)–3(F)). For instance, there were only 20.8 and 11.2% normal embryos at 11 d after pollination in “Jinsenianhua” × “Qinhuaihuadeng” and “Qinhuaihuadeng” × “Jinsenianhua”, respectively (Table 2; Figures 3(G), 3(H)). The percentage of normal embryos at each developmental stage in the cross of “Jinsenianhua” × “Qinhuaihuadeng” was much higher than that at the corresponding time in the other cross.

### 3.4. Seed Set of the Two Lotus Crosses

Seed set in the “Jinsenianhua” × “Qinhuaihuadeng” cross was 17.9%, which was more than twice that in the “Qinhuaihuadeng” × “Jinsenianhua” cross (8.0%; Table 3). At 25 d after artificial pollination, most normal seeds were nearly mature (Figure 3(E)) and normal seeds became dark brown and were completely mature at approximately 30 d after pollination (Figure 3(F)).

## 4. Discussion

Seed production of crops is usually closely related to pollen viability [14–18]. If pollen grains with low viability are pollinated onto stigmas of female parents in crop crosses, the probabilities of pollination failure will increase. As a consequence, seed set will be low and breeding efficiency will be reduced [19, 20]. In crosses between rice subspecies, the low pollen viability of male parents was the main factor leading to low fecundity of the crosses [20]. Similar phenomena have been observed in chrysanthemum and soybean [21, 22]. In the present study, the highest pollen viabilities of the two cultivars were only 20.6% and 15.7%, respectively (Figure 1). It initially seemed that poor pollen viability may have some negative effects on seed set of the two lotus crosses; however, this is not true for the following reasons. The percentages of normal embryos at 1 d after artificial pollination were 55.0 and 21.9% for “Jinsenianhua” × “Qinhuaihuadeng” and “Qinhuaihuadeng” × “Jinsenianhua”, respectively (Table 2). In addition, the corresponding highest pollen viabilities of male plants were 15.7 and 20.6% in the two crosses (Figure 1). Furthermore, the fertilization rate of ovules not only has a close relationship with pollen viability, but also is more closely related to the absolute quantity of pollen grains germinating on stigmas [13, 22]. These suggest that the large difference in percentages of normal embryos at 1 d after artificial pollination in the two crosses may be attributed to other factors, not to pollen viability. We therefore speculated that low pollen viability may not be the main factor influencing seed production of the two lotus crosses.

Whether pollen and stigma can identify each other is also an important factor affecting seed set of plant crosses [23–28]. If pollen and pistil fail to recognize each other normally, most pollen grains may fail to germinate or germinate abnormally even they have very high viability. As a consequence, low pistil receptivity will result in failure of fertilization and low fecundity in the crosses. In this study, the numbers of pollen grains germinated per lotus stigma reached a peak at 4 h after artificial pollination of 63.0 and 17.9 in “Jinsenianhua” × “Qinhuaihuadeng” and “Qinhuaihuadeng” × “Jinsenianhua”, respectively. The 17.9 germinated pollen grains per stigma in “Qinhuaihuadeng” × “Jinsenianhua” may not have been sufficient to fertilize one pistil. The possible reasons may be that most pollen tubes had abnormalities and few pollen tubes could grow toward the embryo sac along the long style. Finally, most pollen tubes failed to reach the embryo sac and only a few pollen tubes entered the embryo sac. The low percentage of normal embryos (21.9%) at 1 d after artificial pollination further supports this explanation. However, 63.0 germinated pollen grains in “Jinsenianhua” × “Qinhuaihuadeng” may be sufficient to fertilize a pistil, as confirmed by the high percentage of normal embryos (55.0%) at 1 d after artificial pollination. Therefore, low pistil receptivity may be partly responsible for low seed set in “Qinhuaihuadeng” × “Jinsenianhua”, while seed set in “Jinsenianhua” × “Qinhuaihuadeng” was less negatively influenced by the interaction between pollen and stigma.

Embryo development is a further factor influencing seed set, and embryo abortion usually leads to low seed set [10, 19, 29, 30]. For instance, Sun et al. [11] reported that embryo abortion was a critical factor resulting in the failure of the interspecies cross between *D. grandiflorum* “Yuhuaxingchen” and *C. nankingense* and a main factor leading to low seed set of *D. grandiflorum* “Yuhuaxingchen” and *D. zawadskii*. Deng et al. [31] found that a postfertilization barrier, that is, abortion of many embryos at various developmental stages before maturation significantly reduced fecundity between *Chrysanthemum* and *Ajania*. Similarly, in the interspecies cross between *P. vulgaris* and *P. coccineus*, Ndoutoumou et al. [10] also found that embryo abortion after fertilization was a key factor resulting in the failure of this cross. In the present study, many embryos aborted during their developmental processes in the two crosses. There were 55.0 and 21.9% normal embryos at 1 d after pollination in “Jinsenianhua” × “Qinhuaihuadeng” and “Qinhuaihuadeng” × “Jinsenianhua”, respectively; however, corresponding values at 20 d after pollination decreased to 20.8 and 11.2%. Such results clearly indicate that embryo abortion was a main factor dramatically reducing seed set of both lotus crosses.

Seed set in “Jinsenianhua” × “Qinhuaihuadeng” was 17.9%, about 2.2 times that in “Qinhuaihuadeng” × “Jinsenianhua” with 8.0%. Such a large difference in seed set of the two crosses may be largely due to difference in pistil receptivity. For example, there was no significant difference in the highest pollen viability of the two lotus cultivars. In addition, there were 63.0 germinated pollen grains in “Jinsenianhua” × “Qinhuaihuadeng”, about 3.7 times of that in “Qinhuaihuadeng” × “Jinsenianhua” with 17.2. Moreover, the percentages of normal embryos at 1 d after pollination in the two crosses were 55.0 and 21.9%, respectively, A 2.35-fold discrepancy. Therefore, the difference in percentages of normal embryos at 1 d after pollination in the two crosses may be mainly attributed to the difference in the number of germinated pollen grains. Taken together, these results suggest that a large difference in pistil receptivity may be mainly responsible for the large difference in seed set of the two crosses. However, the reasons for the differences in pistil receptivity in the two crosses remain unclear. In addition, female cytoplasm may also have some effects on seed set of the reciprocal crosses. 

In conclusion, we systematically investigated the possible factors influencing fecundity of two lotus crosses, mainly including pollen viability, pistil receptivity, and embryo development. There were three findings of note. Firstly, low pollen viability had no significant effects on seed set of the lotus crosses. Secondly, low pistil receptivity and embryo abortion were two main factors causing low seed set in “Qinhuaihuadeng” × “Jinsenianhua”, and the low fecundity of “Jinsenianhua” × “Qinhuaihuadeng” was mainly attributable to embryo abortion. Thirdly, the large difference in seed set in the two crosses was largely due to the large difference in pistil receptivity of the two crosses. These results suggest that special pollination methods and embryo rescue techniques may be effective in overcoming reproductive barriers and enhancing breeding efficiency in lotus crosses in future.

## Figures and Tables

**Figure 1:** Viabilities of pollen grains collected at different times.

**Figure 2:** Pollen grains and pollen tubes on stigmas at 4 h after pollination and anatomical structure of young embryos. (A): Many pollen grains germinated on stigmas in “Jinsenianhua” × “Qinhuaihuadeng”. (B): A few pollen grains germinated on stigmas in “Qinhuaihuadeng” × “Jinsenianhua”. (C and D): Some abnormal pollen tubes in “Qinhuaihuadeng” × “Jinsenianhua”. (E): SEM micrograph of an abnormal pollen tube in “Qinhuaihuadeng” × “Jinsenianhua”. (F): SEM micrograph of a normal pollen tube in “Jinsenianhua” × “Qinhuaihuadeng”. (G): A normal globular embryo at 1 d after artificial pollination. (H): A normal heart embryo at 2 d after artificial pollination. Abbreviations: E (endosperm), Ge (globular embryo), He (heart embryo), I (integument), Pc (papilla cell), Pg (pollen grain), and Pt (pollen tube).

**Figure 3:** The morphology of lotus ovary, seed, and seed pod at different times after pollination. (A): Normal ovaries at 5 d after pollination. (B): Abnormal ovaries at 5 d after pollination. (C): Normal ovaries at 11 d after pollination. (D): Abnormal ovaries at 11 d after pollination. (E): Seeds at 25 d after pollination. (F): Seeds at 30 d after pollination. (G): Lotus seed pod at 11 d after pollination in “Jinsenianhua” × “Qinhuaihuadeng” (asterisks indicate normal seeds). (H): Lotus seed pod at 11 d after pollination in “Qinhuaihuadeng” × “Jinsenianhua” (asterisks indicate normal seeds). Abbreviations: Ao (abnormal ovary); No (normal ovary).

**Table 1:** Number of pollen grains germinating on stigma after pollination.

Time after pollination (h)	Number of pollen grains germinating per stigma in the two crosses	
	“Jinsenianhua” × “Qinhuaihuadeng”	“Qinhuaihuadeng” × “Jinsenianhua”
0.5	16.4 ± 1.1	11.2 ± 2.6
1	20.2 ± 2.6	13.6 ± 2.1
2	34.4 ± 3.4	15.0 ± 2.2
4	63.0 ± 6.8	17.2 ± 1.9
6	41.6 ± 3.9	14.2 ± 1.6
8	24.8 ± 2.6	10.0 ± 1.6
10	20.4 ± 3.2	8.2 ± 1.5
12	13.8 ± 2.9	7.4 ± 1.7

**Table 2:** Number of normal and abnormal embryos at different days after pollination.

Crosses	Days after pollination	Developmental stages	Percentage of normal embryo (%)
“Jinsenianhua” × “Qinhuaihuadeng”	1	Globular embryo	55.0 ± 6.3
	2	Heart embryo	37.5 ± 4.5
	4	Cotyledon embryo	29.8 ± 4.2
	6		25.5 ± 3.7
	8		21.6 ± 3.1
	11		20.8 ± 3.3
“Qinhuaihuadeng” × “Jinsenianhua”	1	Globular embryo	21.9 ± 2.9
	2	Heart embryo	14.7 ± 1.8
	4	Cotyledon embryo	12.9 ± 1.6
	6		12.0 ± 1.5
	8		12.5 ± 1.2
	11		11.2 ± 1.4

**Table 3:** Seed set of the two lotus crosses.

Crosses	Seed set (%)
“Jinsenianhua” × “Qinhuaihuadeng”	17.9 ± 2.5
“Qinhuaihuadeng” × “Jinsenianhua”	8.0 ± 1.4

## References

[1] Han YC, Teng CZ, Chang FH (2007). Analyses of genetic relationships in *Nelumbo nucifera* using nuclear ribosomal ITS sequence data, ISSR and RAPD markers. *Aquatic Botany*.

[2] Han YC, Teng CZ, Wahiti GR, Zhou MQ, Hu ZL, Song YC (2009). Mating system and genetic diversity in natural populations of *Nelumbo nucifera* (Nelumbonaceae) detected by ISSR markers. *Plant Systematics and Evolution*.

[3] Guo HB (2009). Cultivation of lotus (*Nelumbo nucifera* Gaertn. ssp. *nucifera*) and its utilization in China. *Genetic Resources and Crop Evolution*.

[4] Huang GZ (1982). Studies on the biology of anthesis and the technique of artificial pollination of the lotus (*Nelumbo nucifera* Gaertn.). *Acta Horticulturae Sinica*.

[5] Wang QC, Zhang XY (2005). *Chinese Lotus*.

[6] Jiang L, Chen FD, Cui NX, Gu JJ (2008). Study on seed setting of hybridization, selfing and open pollination of six cultivars of *Nelumbo nucifera*. *Acta Agricuturae Shanghai*.

[7] Chen XL, Bao JZ, Liu CG, Cao H, Zhai JQ (2004). Preliminary study on irradiation breeding of ornamental lotus. *Acta Agriculturae Nucleatae Sinica*.

[8] Li YH, Pan YZ, Chen YQ (2008). Advance in researches on the genetic diversity of *Nelumbo nucifera*. *Journal Sichuan Forestry Science and Technology*.

[9] Marta AE, Camadro EL, Díaz-Ricci JC, Castagnaro AP (2004). Breeding barriers between the cultivated strawberry, *Fragaria* × *ananassa*, and related wild germplasm. *Euphytica*.

[10] Ndoutoumou PN, Toussaint A, Baudoin JP (2007). Embryo abortion and histological features in the interspecific cross between *Phaseolus vulgaris* L. and *P. coccineus* L. *Plant Cell, Tissue and Organ Culture*.

[11] Sun CQ, Chen FD, Teng NJ, Liu ZL, Fang WM, Hou XL (2010). Factors affecting seed set in the crosses between *Dendranthema grandiflorum* (Ramat.) Kitamura and its wild species. *Euphytica*.

[12] Teng N, Chen T, Jin B (2006). Abnormalities in pistil development result in low seed set in *Leymus chinensis* (Poaceae). *Flora*.

[13] Jin B, Wang L, Wang J (2010). The structure and roles of sterile flowers in *Viburnum macrocephalum* f. *keteleeri* (Adoxaceae). *Plant Biology*.

[14] Dafni A, Firmage D (2000). Pollen viability and longevity: practical, ecological and evolutionary implications. *Plant Systematics and Evolution*.

[15] Wilcock C, Neiland R (2002). Pollination failure in plants: why it happens and when it matters. *Trends in Plant Science*.

[16] Hu SY (2005). *Reproductive Biology of Angiosperms*.

[17] Li H, An S, Zhi Y (2008). Protogynous, pollen limitation and low seed production reasoned for the dieback of Spartina anglica in coastal China. *Plant Science*.

[18] Park NI, Yeung EC, Muench DG (2009). Mago Nashi is involved in meristem organization, pollen formation, and seed development in Arabidopsis. *Plant Science*.

[19] Meng JL (1977). *Genetics of Plant Reproduction*.

[20] Fan FL, Tang XR (2002). Recent progress on the study of the fecundity of cross rice between subspecies. *Crop Research*.

[21] Zhao LM, Sun H, Huang M, Wang SM, Wang YQ (2004). The relationship between seed setting rate and pollen sterility rate for soybean. *Soybean Science*.

[22] Sun CQ, Huang ZZ, Wang YL (2011). Overcoming pre-fertilization barriers in the wide cross between *Chrysanthemumgrandiflorum* (Ramat.) Kitamura and *C. nankingense* (Nakai) Tzvel. by using special pollination techniques. *Euphytica*.

[23] Mazzucato A, Olimpieri I, Ciampolini F, Cresti M, Soressi GP (2003). A defective pollen-pistil interaction contributes to hamper seed set in the *parthenocarpic* fruit tomato mutant. *Sexual Plant Reproduction*.

[24] Huang Z, Zhu J, Mu X, Lin J (2004). Pollen dispersion, pollen viability and pistil receptivity in *Leymus chinensis*. *Annals of Botany*.

[25] Aliyu OM (2007). Pollen-style compatibility in cashew (*Anacardium occidentale* L.). *Euphytica*.

[26] Lee CB, Page LE, McClure BA, Holtsford TP (2008). Post-pollination hybridization barriers in *Nicotiana* section *Alatae*. *Sexual Plant Reproduction*.

[27] Ganesh Ram S, Hari Ramakrishnan S, Thiruvengadam V, Kannan Bapu JR (2008). Prefertilization barriers to interspecific hybridization involving *Gossypium hirsutum* and four diploid wild species. *Plant Breeding*.

[28] Wheeler MJ, De Graaf BHJ, Hadjiosif N (2009). Identification of the pollen self-incompatibility determinant in *Papaver rhoeas*. *Nature*.

[29] Mallikarjuna N, Saxena KB (2002). Production of hybrids between *Cajanus acutifolius* and *C. cajan*. *Euphytica*.

[30] Datson PM, Murray BG, Hammett KRW (2006). Pollination systems, hybridization barriers and meiotic chromosome behaviour in Nemesia hybrids. *Euphytica*.

[31] Deng Y, Chen S, Teng N (2010). Flower morphologic anatomy and embryological characteristics in *Chrysanthemum multicaule* (Asteraceae). *Scientia Horticulturae*.

